# XuefuZhuyu decoction protected cardiomyocytes against hypoxia/reoxygenation injury by inhibiting autophagy

**DOI:** 10.1186/s12906-017-1822-0

**Published:** 2017-06-19

**Authors:** Xiaowen Shi, Haiyan Zhu, Yuanyuan Zhang, Mingmei Zhou, Danli Tang, Huamin Zhang

**Affiliations:** 1 Center for Chinese Medical Therapy and Systems Biology, Shanghai University of Traditional Chinese Medicine, Shanghai, 201203 People’s Republic of China; 2 Department of Microbiological & Biochemical Pharmacy, School of Pharmacy, Fudan University, 826 Zhangheng Road, Shanghai, 201203 People’s Republic of China; 3 Department of Pharmacology, West China School of Preclinical and Forensic Medicine, Sichuan University, Chengdu, 610041 People’s Republic of China; 4 Institute of Information on Traditional Chinese Medicine, China Academy of Chinese Medical Sciences, No.16, Nanxiao Road, Dongzhimen, Beijing, 100700 People’s Republic of China

**Keywords:** XuefuZhuyu decoction, Hypoxia/reoxygenation, Autophagy, Ischemic/reperfusion, mTOR

## Abstract

**Background:**

XuefuZhuyu decoction (XFZY) is a well-known traditional Chinese herbal medicine for the treatment of various cardiovascular diseases, such as unstable angina pectoris and myocardial ischemia-reperfusion injury. However, the mechanism by which XFZY contributes to the amelioration of cardiac injury remains unclear.

**Methods:**

H9C2 cells were cultured under the hypoxic condition for 10 h and reoxygenated for 2 h. In the presence of various concentrations of XFZY for 12 h, the cell viability was measured by MTT assay. The protective effect of XFZY in hypoxia/reoxygenation (H/R) cell model was confirmed by measuring the amount of LDH released into the extracellular fluid. Cell apoptosis was measured by western blotting. The autophagy level of H9C2 cells and the correlative pathway were determined by transmission electron microscopy, Cyto-ID® Autophagy Detection Kit, and western blotting.

**Results:**

In this study, we investigated the effects of XFZY on H/R induced cardiac injury. The results showed that treatment with XFZY significantly inhibited autophagy induced by H/R, with decreased formation of autophagosomes as well as the expression of LC3-II/LC3-I ratio and Beclin 1 after H/R. Importantly, inhibition of autophagy by XFZY resulted in enhanced cell viability and decreased apoptosis. XFZY also inhibited the activation of AMPK and upregulated the phosphorylation of mammalian target of Rapamycin (mTOR).

**Conclusions:**

The cardioprotective effects of XFZY during H/R were mediated by inhibiting autophagy via regulating AMPK-mTOR signaling pathways.

## Background

XuefuZhuyu decoction (XFZY) is a well-known traditional Chinese herbal medicine recorded in the *Yi Lin Gai Cuo* compiled by Qing-ren Wang in the Qing dynasty (AD 1830). XFZY has multiple effects such as anti-inflammation [1], antioxidant and drug-metabolizing enzymes [2] and angiogenesis modulation [3]. XFZY is very effective in the treatment of various cardiac diseases, such as myocardial fibrosis [4], hypertension [5], unstable angina pectoris [6], atherosclerosis [7] and myocardial ischemia-reperfusion injury [8]. We have recently found that XFZY could ameliorate hypoxia-reoxygenation (H/R) induced cardiac injury. In this study, we established an H/R-induced cardiomyocyte injury model that caused the death of cardiomyocyte H9C2 cells and investigated the mechanisms by which XFZY contributed to the amelioration of cardiomyocyte apoptosis.

Ischemia-reperfusion (I/R) induced myocardial injury is considered to be the main cause of acute myocardial infarction, which is mainly caused by the restoration of blood flow to the ischemic myocardium. There is increasing evidence that oxidative stress, apoptosis, Ca^2+^ overload, and autophagy is involved in this process [9, 10]. Autophagy is a major catabolic mechanism by which mammalian cells degrade and recycle macromolecules and organelles at the basal level under normal conditions, contributing to maintaining intracellular homeostasis by removing protein aggregates and damaged organelles. However, autophagy plays quite different roles in the myocardial ischemia and reperfusion. During ischemia, a low level of ATP can activate AMP-activated protein kinase (AMPK)-mammalian target of Rapamycin (mTOR) pathway, which leads to autophagy initiation and cardioprotection; while during reperfusion, increased reactive oxygen species could result in the upregulation of Beclin 1 and thus the death of autophagic cells [11].

In this study, low-toxicity XFZY that could be absorbed by small intestine was used as an alternative to drug-containing serum and extraction solution, and then we investigated whether autophagy was involved in XFZY induced cardiomyocyte protection. Our results clearly showed that the treatment with XFZY resulted in a lower autophagic level than negative controls. More importantly, the inhibition of autophagy by XFZY significantly rescued cell viability and decreased apoptosis in H9C2 cells. We also investigated the relationship between autophagy and its upstream regulators. Our results provided a new mechanistic insight into the role of XFZY against H/R-induced cardiomyocyte injury.

## Methods

### Preparation of XFZY

XFZY was provided by Beijing Tongrentang (Bozhou) Prepared Slices of Chinese Crude Drugs Co., Ltd., which consisted of 11 herbs, as shown in Table 1. These herbs were macerated for 2-3 h with 4 L of distilled water and decocted for 40 min. The filtrate was collected and the residue was decocted again for 40 min with 2.5 L of distilled water for the collection of filtrate again. The two filtrates were combined and then condensed to 4.3 g/ml. The volume of XFZY solution was diluted to 600 ml with Tyrode’s buffer solution (NaCl 8.00 g, KCl 10.28 g, NaHCO_3_ 1.00 g, NaH_2_PO_4_ 0.05 g, MgCl_2_ 0.10 g, CaCl_2_ 0.20 g, and glucose 1.00 g; pH 7.4).

**Table 1:** The composition of XFZY

Drug name	Latin name	Amount (g)
Chinese Angelica	*Angelica sinensis *(Oliv.)Diels	9.0
Dried Rehmannia root	*Rehmannia glutinosa* Libosch	9.0
Peachseed	* Prunu persica* (L.) Batsch	12.0
Safflower	*Carthamus tinctorius* L.	9.0
Radix Paeoniae Rubra	*Paeonia Lactiflora *Pall.	6.0
Radix Bupleuri	*Bupleurum chinense* DC.	3.0
Fructus Aurantii	*Citrus aurantium *L.	6.0
Licorice Roots Northwest Origin	*Glycyrrhiza uralensis *Fisch.	6.0
Balloon Flower	*Platycodon grandiflorum* (Jacq.)A.DC.	4.5
Ligusticum wallichii	*Ligusticum chuanxiong* Hort.	4.5
Cyathula Officinalis	*Achyranthes bidentata* Blume	9.0

Male Sprague-Dawley Rats were maintained under fasting conditions for 12 h before the experiment. Their small intestines were quickly removed under anesthesia, washed with Tyrode buffer solution (0 °C) and cut into four segments of 14 cm each. Each segment was turned inside-out and ligated to form a sac at one end. Then, the sac was filled with Tyrode buffer and incubated in Magnus’bath for 5 min to reach equilibrium. The buffer was exchanged with XFZY solution (25 mL), and the segment was maintained at 37 °C in a 95%O_2_/5%CO_2_ atmosphere. Serosalside solutions containing absorbed constituents (2.5 ml) were drained into tubes after 2 h. XFZY was filtered with a microfiltration membrane (0.22 μm) and stored at -20 °C.

### Chromatographic analysis of XFZY

High-performance liquid chromatography (HPLC) was performed on an Agilent 1290 UPLC system (Agilent Technologies, Waldbronn, Germany) connected to an Agilent 6520 Q-TOF mass spectrometer (Agilent Corporation, Santa Clara, CA, USA) via an ESI interface. Acetonitrile and methanol (HPLC grade) were purchased from Fisher Scientific (Pittsburg, PA, USA). Formic acid (HPLC grade) was purchased from Damao (Tianjin, China). Water for HPLC was purified by a Milli-Q water purification system (Millipore, Bedford, MA, USA), and polytetrafluoroethylene (PTFE) membranes of 0.2 μm purchased from Millipore (Bedford, MA, USA) were used for processing samples.

The separation was carried out on a ZORBAX SB-C18 column (100 mm × 4.6 mm, 1.8 μm particle size, Agilent) at 50 °C with a flow rate of 0.4 mL/min. The mobile phase was a mixture of 0.1% formic acid-water (A) and acetonitrile (B). The gradient program of the mobile phase was as follows: 0–2 min, 5–15% B; 2–5 min, 15–25% B; 5–7 min, 25–31% B; 7–9 min, 31–40% B; 9–12 min, 40–75% B; and 12–15 min, 75–95% B. The injection volume was 2 μL.

The acquisition parameters of Hybrid quadrupole time-of-flight mass spectrometry (QTOF) were as follows: drying gas (N_2_) flow rate, 10.0 L/min; drying gas temperature, 350 °C; nebulizer gas pressure, 40 psi; capillary voltage, 4500 V; fragmentor voltage, 150 V; skimmer voltage, 65 V; and octopole RF, 750 V. The sample was analyzed in both positive and negative ion modes to provide complementary information for structural identification.

The quasi-molecular ions [M − H]^−^ and [M + H]^+^ were selected as the precursor ions and subjected to target-MS/MS analyses. The collision energy (CE) was set at 15-40 V and the mass range was recorded from m/z 100 to 1000.

### Cell culture

Rat H9C2 cells obtained from Shanghai Institutes for Biological Sciences, Chinese Academy of Sciences, were cultured in high glucose DMEM (Corning, USA) and 10% heat-inactivated fetal bovine serum (Invitrogen, San Diego, CA, USA) supplemented with 100 U/mL penicillin and 100 g/mL streptomycin (Beyotime Institute of Biotechnology, Haimen, China) at 37 °C in a 95% air/5% CO_2_ atmosphere. The medium was replaced every 2–3 days, and cells were subcultured or subjected to experimental procedures at 80–90% confluence.

### H/R injury model in vitro

H/R injury model in vitro was established as previously described [12]. H9C2 cells were incubated in the hypoxic/ischemic chamber (Anaerocult® A mini, Merck) in serum-free and low-glucose DMEM at 37 °C for 10 h in a humidified atmosphere of 5% CO_2_ and 95% nitrogen, and then incubated with fresh medium and restored to 95% nitrogen/5% CO_2_ for 2 h reoxygenation. At the onset of hypoxia, cardiomyocytes were randomly treated with 4.5, 9 and 18 mg/ml XFZY with Tyrode buffer as a vehicle, respectively, and, H9C2 cells cultured under normal conditions in a CO_2_ incubator served as negative controls. At the same time, cell model of starvation/rapamycin-induced autophagy was established in H9C2 cells. Cells were incubated in serum-free medium or with rapamycin (500 nm) in the presence or absence of XFZY for 10 h, and the protein expression of LC3 (normalized to that of GAPDH) was assayed.

### Cell viability assay

Cell viability was determined by MTT cytotoxicity assay. Cells were seeded in 96-well plates at a concentration of 2 × 10^4^ cells/well. After the cells adhered, the medium was replaced with serum-free and low-glucose DMEM (Thermo Fisher Scientific, Beijing, China) or various concentrations (4.5, 9, 18, 36, and 72 mg/ml) of XFZY in low glucose DMEM. After incubation for 48 h, the cytotoxicity of XFZY was assayed by MTT. Cells in each group were cultured under hypoxic conditions for 10 h and reoxygenated for 2 h (H10/R2). Cells were incubated with MTT (0.5 mg/ml) for 4 h at 37 °C, and then the supernatants were carefully removed, and the formazan crystal was dissolved in DMSO and quantified spectrophotometrically at 570 nm. The reduction in optical density was considered to be the decrease in cell viability.

### Measurement of lactate dehydrogenase (LDH) release in culture supernatants

Cell injury was confirmed by measuring the amount of LDH released into the extracellular fluid from damaged cells after H10/R2 injury. H9C2 cells were plated in 96-well plates as described in the MTT assay. Ten hours later, the amount of LDH was detected by an LDH assay kit (Beyotime Biotechnology, Haimen, China) according to the manufacturer’s instruction with a microplate Reader at 450 nm.

### Transmission electron microscopy

H9C2 cells were fixed with 2% glutaraldehyde for 15 min and then fixed in 2% glutaraldehyde with 0.1 M Na-Cacodylate/HCl (pH 7.4) for 30 min. They were washed three times with 0.2 M Na Cacodylate/HCl (pH 7.4), fixed with 1% OsO_4_–0.15 M Na Cacodylate/HCl (pH 7.4) for 30 min, and then dehydrated in a growing gradient of ethanol and finally polymerized at 60 °C for 48 h. Samples were cut and analyzed with a JEM 1230 transmission electron microscope (JEOL, Peabody, MA).

### Western blot analysis

H9C2 cells were harvested, washed twice with cold phosphate-buffered saline (PBS), and kept in RIPA lysis buffer (Beyotime Institute of Biotechnology, Jiangsu, China) for 30 min on ice. Then, the lysates were centrifuged, and the supernatants were collected. The protein concentration was examined by the bicinchoninic acid (BCA) method. Equivalent amounts of protein were separated by sodium dodecyl sulfate-polyacrylamindegelelectrophoresis (SDS-PAGE) and then transferred to poly-vinylidene fluoride membranes. The membranes were blocked in Tris-buffered saline and Tween 20 (TBST) containing 3% bovine serum albumin (BSA) for 1 h at room temperature, and incubated with the primary antibodies at 4 °C overnight and then with the second antibody conjugated with horseradish peroxidase for 2 h at room temperature. Then, the membranes were washed in TBST and the signals were visualized using an enhanced chemiluminescent detection kit (Pierce, Rockford, IL). Densitometric values of protein bands were quantified by the IQuantTL software (GE Healthcare, USA).

### Confocal immunofluorescence

H9C2 cells were seeded into clear bottom imaging tissue culture plates (NEST Biotechnology Co., Ltd., Jiangsu, China). After 24 h of incubation, cells were treated with an equal volume of the vehicle with or without XFZY (18, 9, or 4.5 mg/mL) for another H10/R2 incubation. Cells were treated with Cyto-ID Autophagy Detection Kit (Enzo Life Sciences, Inc.) according to the manufacturer’s instruction. Briefly, cells were washed twice with assay buffer and stained with Cyto-ID and Hoechst 33,342 at 37 °C for 30 min. After incubation, cells were washed again with 1 × assay buffer and immediately analyzed with an Olympus fluorescence microscope.

### Statistical analysis

All statistical analyses were performed using GraphPad Prism 5. The results were expressed as mean ± SD. Statistical comparisons were performed using One-way ANOVA, and *P* values <0.05 were considered statistically significant.

## Results

### Chromatographic analysis of XFZY

Generally, the components of the decoction are qualitatively identified by the chemical substances from the involved single herbs. A total of nine compounds were identified or tentatively characterized in XFZY by comparing their characteristic high-resolution mass data with that of previous studies [13–16]. The mass error for molecular ions of all identified compounds was within ± 6 ppm, and the total ion chromatograms in negative and positive ion modes were displayed in Fig. 1.

**Fig. 1:** Typical total ion chromatograms obtained from XFZY in the positive **a** and negative modes **b**. Hydroxysafflor yellow A (1), Paeoniflorin (2), Ferulic acid (3), Liquiritoside (4), Anhydrosafflor yellow B (5), Naringin (6), Hesperidin (7), Neohesperidin (8), and Glycyrrhizic acid (9) were identified or tentatively characterized in XFZY

### XFZY protected against H/R injury in cardiomyocytes

In order to determine whether XFZY protected cardiomyocytes against H/R injury, we first examined the toxicity of XFZY to H9C2 cells under normoxic conditions, and then examined that of XFZY after H/R treatment at the toxic concentration. As shown in Fig. 2, 4.5, 9 and 18 mg/ml of XFZY had no toxic effects on H9C2 cells under normoxic conditions, while XFZY exhibited toxicity on H9C2 cells at 36 and 72 mg/ml under normoxic conditions. H/R treatment triggered significant morphological changes of H9C2 cells with reduced cell viability and leakage of cardiac enzymes, which could be reversed by 4.5, 9 and 18 mg/ml of XFZY (Fig. 3a and b). And H9C2 cells treated with 4.5, 9 and 18 mg/ml of XFZY showed no significant morphological changes compared to negative controls. Thus, XFZY protected H9C2 cells against the H/R injury.

**Fig. 2:** Effects of XFZY on cardiomyocyte viability. Myocardial H9C2 cells were subjected to normoxia for 24 h and then incubated with MTT for 4 h at 37 °C. The results were expressed as mean ± SD. ***p < 0.001 vs Control group

**Fig. 3:** Protection of XFZY against H/R-induced cardiomyocyte injury. Myocardial H9C2 cells were incubated with different concentrations of XFZY under hypoxia for 10 h and reoxygenated for 2 h. **a** After H/R, cells were observed under an optical microscope for morphological changes; **b** LDH released from H9C2 cells was assayed after H/R injury. The results were expressed as mean ± SD. ***p < 0.001 vs H/R group; ^*###*^ *p < 0.001* vs Vehicle group. Vehicle: normoxia; H/R: hypoxia/reoxygenation

### XFZY inhibited apoptosis of cardiomyocytes induced by H/R injury

To further explore the protection of XFZY against H/R-induced injury, apoptosis protein levels were examined in H9C2 cells treated with H/R and/or XFZY. Figure 4 clearly showed that H/R induced cleavage of the apoptosis-related protein, poly ADP-ribose polymerase (PARP) in H9C2 cells, indicating the activation of apoptosis. However, XFZY attenuated the expression of cleaved PARP, suggesting XFZY to inhibit apoptosis of cardiomyocytes induced by H/R injury. Furthermore, H9C2 cells treated with H10/R2 and XFZY showed a lower RARP activity than that treated only with H10/R2. Thus, XFZY prevented H/R-induced apoptosis in cardiac cells.

**Fig. 4:** XFZY inhibited apoptosis of H9C2 cells subjected to H/R. H9C2 cells were treated with XFZY under H10/R2, and the changes in RAPA expression were examined by western blot. The data were represented as mean ± SD of three independent experiments. Tubulin protein was used as a loading control. *p < 0.05, **p < 0.01 vs H/R group; ^*##*^ *p < 0.01* vs Vehicle group

### XFZY inhibited autophagy of cardiomyocytes induced by H/R injury

In order to determine the effect of XFZY on autophagy of cardiomyocytes induced by H/R injury, we analyzed the expression of autophagy marker proteins at different time points during H10/R2. The results clearly showed that the expression of LC3-II increased gradually during hypoxia and reached a peak after reoxygenation for 2 h (Fig. 5). We speculated that inhibition of autophagosomes formation by XFZY could contribute to the survival of H9C2 cells under H/R conditions. Then, we observed ultra-structural changes in H9C2 cells after H/R by transmission electron microscopy and analyzed the expression of autophagy marker proteins LC3-I/II in H9C2 cells under normoxic and H/R conditions by western blot. Figure 6a and c showed that H/R resulted in a significant increase in LC3-II expression and autophagosomes formation, while XFZY inhibited the transform of LC3-I to LC3-II and the number of autophagosomes compared to H9C2 cells cultured under H/R conditions. H/R also led to the accumulation of autophagic fluorescence (green fluorescence) in H9C2 cells (Fig. 6b). The quantitative analysis of relative autophagic fluorescence intensity showed that XFZY inhibited the continuous accumulation of autophagosomes and the transform of LC3-I to LC3-II after H10/R2. Thus, autophagy could be triggered by H/R in H9C2 cells, and XFZY significantly inhibited the accumulation of autophagosomes.

**Fig. 5:** The expression of autophagy marker proteins at different time points of H10/R2. H9C2 cells were cultured under hypoxia for 0 h (H0), 2 h (H2), 4 h (H4), 6 h (H6), 8 h (H8) and 10 h (H10), and reoxygenated for 2 h (H10/R2), respectively. The expression of LC3, an autophagy marker, was assayed. The data were represented as mean ± SD of three independent experiments. Tubulin protein was used as a loading control. ** p < 0.05 vs H0 group

**Fig. 6:** Effect of XFZY on H/R-induced autophagy in H9C2 cells. **a** Ultra-structural changes in H9C2 cells after H/R by transmission electron microscopy (10,000×). **b** Autophagic vacuoles were analyzed by confocal microscopy. Cells were plated in cell culture dishes with a glass bottom. After XFZY treatment, cells were concurrently stained with Cyto-ID Green dye and Hoechst33342 and detected by confocal microscopy. **c** Protein expression of LC3-II was determined by Western blot. The results were expressed as mean ± SD. ***p < 0.001, **p < 0.01vs H/R group; ^*###*^ *p < 0.001* vs Vehicle group

### MAPK/mTOR signaling pathway was involved in the inhibition of autophagy of cardiomyocytes induced by H/R injury

To determine the molecular mechanism of autophagy of cardiomyocytes induced by H/R injury, expressions of a series of upstream proteins, such as AMPK, beclin1, and mTOR, were evaluated. We found that XFZY decreased the phosphorylation of AMPK, beclin1, and LC3-II, but increased that of mTOR, which indicated H/R-induced autophagy to be mediated by inhibition of mTOR expression (Fig. 7). Our results also indicated that inhibition of AMPK could relieve H/R-induced autophagy and protect against cardiac injury.

**Fig. 7:** XFZY inhibited autophagy through AMPK-mTOR pathway in H9C2 cells subjected to H/R. H9C2 cells were treated with XFZY under H10/R2. Expressions of AMPK **a**, beclin-1 **b** and mTOR **c** were examined by western blot. The data were expressed as the means ± SD of three independent experiments. ***p < 0.01, **p < 0.01, *p < 0.05 vs H/R group; ^*###*^ *p < 0.001,* ^*##*^ *p < 0.01* vs Vehicle group

### XFZY inhibited starvation/rapamycin-induced autophagy in cardiomyocytes

Since H/R-induced autophagy could be modulated by inhibiting mTOR signaling in H9C2 cells and partly rescued by XFZY, we hypothesized that XFZY may act as an autophagy inhibitor during energy deprivation and rapamycin-induced autophagy by regulating p-mTOR. Thus, we analyzed the inhibitory effect of XFZY on starvation and rapamycin-induced autophagy. As shown in Fig. 8, the LC3-II/LC3-I to GAPDH ratio was significantly increased by starvation and rapamycin in H9C2 cells, and XFZY inhibited starvation and Rapamycin-induced autophagy at 4.5, 9, and 18 mg/ml. Thus, XFZY inhibited the upstream of the AMPK-mTOR pathway.

**Fig. 8:** XFZY inhibited starvation/rapamycin-induced autophagy in H9C2 cells. **a** Cells were incubated in serum-free medium in the absence or presence of XFZY for 10 h, and the protein expression of LC3 was assayed. **b** Cells were incubated with rapamycin (500 nm) in the absence or presence of XFZY for 10 h, and the protein expression of LC3 (normalized to that of GAPDH) was assayed. *p < 0.05, **p < 0.01 vs Control group; ^*#*^ *p < 0.05,* ^*##*^ *p < 0.01* vs Vehicle group

## Discussion

We speculated that XFZY could inhibit H/R-mediated autophagosome formation, which contributed to the survival of H9C2 cells under H/R conditions. In this study, we investigated the mechanisms by which XFZY protected myocardial H9C2 cells against H/R injury. The results clearly showed that XFZY enhanced cell survival and inhibited apoptosis of cardiomyocytes induced by H/R injury, and also modulated autophagy by regulating the activity of AMPK-mTOR signaling pathway. H/R is one of the main pathological factors for cell injury. Previous studies have demonstrated that the animal model in which myocardial cells exposed to low ATP and oxygen depletion could imitate the part of the internal environment of I/R to test the mechanism of therapy in vivo [17]. Thus, H9C2 cell models exposed to H/R were used to mimic I/R induced cell injury in vitro, which contributed to developing effective drugs for the treatment of cardiovascular diseases.

Autophagy is considered to be an important cytoprotective mechanism by which excess or damaged organelles are degraded [18]. Mild activation of autophagy can promote the survival of cells, while excessive activation of autophagy can destroy normal proteins and organelles, leading to the death of autophagic cells. Our results showed that excessive autophagy was involved in H/R-induced cardiomyocyte injury, which was inhibited by XFZY due to enhanced viability and inhibition of apoptosis.

Autophagy can be promoted by AMPK, a key energy sensor capable of regulating cellular metabolism to maintain energy homeostasis. Conversely, it could be inhibited by mTOR, a central cell-growth regulator that integrates growth factor and nutrient signals [19]. It has been shown that H/R induced down-regulation of p-mTOR via the AMPK-mTOR pathway, as tuberous sclerosis complex1/tuberous sclerosis complex 2 (TSC1/TSC2) protein complex was the major suppressor of the mTOR signaling in H9C2 cells exposed to H/R. Our study revealed how XFZY regulated the AMPK-mTOR pathway of autophagy, and inhibition of autophagy was helpful for the survival of H9C2 cells exposed to H/R. In the starvation/rapamycin-induced cell model, XFZY decreased the ratio of LC3-II/LC3-I under the conditions of ATP depletion. In another model in which autophagy was induced by rapamycin, XFZY inhibited the ratio of LC3-II/LC3-I by inhibiting the fusion of autophagosomes and lysosomes. Thus, XFZY inhibited autophagy in cells under different conditions, the mechanism of which may be related to the upstream of mTOR pathway. We speculated that AMPK was not the specific target of XFZY in vitro, but XFZY did protect H/R-induced cardiac injury through the mTOR pathway. However, further studies are needed to identify the target and active components of XFZY.

XFZY is a classic traditional Chinese medicine for the treatment of cardiovascular diseases. However, the active components of XFZY remain unidentified. The small intestine is the major absorption site for herbal medicines. XFZY can be absorbed by small intestine in a similar way as that for most traditional Chinese medicines. The constituents of XFZY absorbed by the digestive tract may produce therapeutic effects [20, 21]. In this study, we tested the intestinal absorption of XFZY in H/R cell model to reveal its protective activity on H/R injury [8], and the results clearly showed that the intestinal absorption of Chinese herbs may be a potential approach to study the mechanism of Chinese herb compounds in vitro*.*

XFZY resulted in a delayed apoptosis and highly inhibited autophagy in H9C2 cells exposed to H/R. Previous studies have shown that apoptosis is one of the main factors involved in the ischemic heart diseases, while inhibition of apoptosis is an important therapeutic approach for ischemic heart diseases. Our study showed that inhibition of autophagy contributed to the inhibition of apoptosis, thus indicating that inhibition of autophagy could be a potential approach for the treatment of H/R injury.

## Conclusion

In conclusion, XFZY significantly relieved damage after H/R injury and improved the survival of cardiomyocytes by inhibiting excessive autophagy. The protection of XFZY against H/R-induced cardiomyocyte injury were mediated by inhibiting excessive autophagy via regulating AMPK-mTOR signaling pathways.

## Abbreviations

BCA: Bicinchoninic acid
BSA: Bovine serum albumin
CE: Collision energy
H/R: Hypoxia/reoxygenation
H10/R2: Hypoxic conditions for 10 h and reoxygenation for 2 h
HPLC: High-performance liquid chromatography
I/R: Ischemia-reperfusion
MI/RI: Myocardial ischemia and reperfusion
mTOR: Mammalian target of rapamycin
PBS: Phosphate-buffered saline
PTFE: Polytetrafluoroethylene
SDS-PAGE: Sodium dodecyl sulfate-polyacrylaminde gel electrophoresis
TBST: Tris-buffered saline and Tween 20
XFZY: XuefuZhuyu decoction.
